# Pre-BMI and Lipid Profiles in Association with the Metabolic Syndrome in Pregnancy with Advanced Maternal Age

**DOI:** 10.1155/2022/4332006

**Published:** 2022-07-09

**Authors:** Xinxin Yang, Rui Jiang, Xiuping Yin, Guangya Wang

**Affiliations:** ^1^Department of Endocrinology, Cangzhou Central Hospital, Cangzhou, China; ^2^Department of Neonatology, Cangzhou Central Hospital, Cangzhou, China

## Abstract

We aimed to explore the association of BMI in pre-pregnant women with metabolic syndrome in pregnancy in advanced maternal age. A total of 229 maternal women and 536 maternal women participated in this study. Pregnancy women underwent a 75 g-oral glucose tolerance test and maternal lipid profile test between 24 and 28 weeks. Data about biological and sociodemographic characteristics were recorded for each case. The metabolic equivalent (Met) was 9.6% in the maternal age ≥35 group, 5.4% in the age 20–34 group (*P* = 0.027), and 6.7% in all pregnant women. Results also demonstrated that gestational diabetes mellitus (GDM) and MetS were more likely to appear in the maternal age ≥35 years group than the maternal age 20–34 years group (41.5% vs. 30.6%; *P* = 0.001, 9.6% vs. 5.4%, *P* = 0.027). Risk for preterm delivery and eclampsia were increased with raised MetS (RR 3.434 and RR 1.800); MetS in women aged ≥35 years had the largest area under the curve (AUC) (AUC 0.925, 95% CI 0.885–0.965), and its optimal cutoff point was ≥24.998 kg/m^2^, and the optimal cutoff point for total cholesterol (TC) (AUC 0.686, 95% CI 0.571–.802) predicting MetS was ≥4.955 mmol/l. MetS in pregnancy are associated with the occurrence of preterm delivery and eclampsia, and pre-BMI and TC can predict MetS in the maternal age ≥35 group.

## 1. Introduction

Less research about MetS in pregnant women has been investigated [1–3]. The number of older women with fertility requirements has gradually increased, and pregnant women over the age of 35 have become a reality facing the world. The impact of obesity on maternal MetS, in advanced maternal age, has not been investigated.

Our research was aimed at discussing the associations between BMI in pre-pregnant and metabolic syndrome during gestation in advanced maternal age and exploring the roles of maternal age and lipid profiles in the metabolic syndrome of pregnancy. In addition, we hope to find more evidence to predict metabolic equivalence in pregnant women and to develop better perinatal care in older mothers.

## 2. Materials and Methods

### 2.1. Enrolled Participants

This study enrolled pregnant women during the period from January 2017 to December 2018 in Cangzhou Central Hospital. Women during singleton pregnancy underwent a 75 g oral glucose tolerance test and maternal lipid profile test between 24 and 28 weeks. Women with previous diagnoses of diabetes, hypertension, and dyslipidemia during a singleton pregnancy and women with overt diabetes diagnosed before 20 weeks of pregnancy were excluded.

### 2.2. Information Collection

A questionnaire with information about biological and sociodemographic characteristics was used for each case. These data included prepregnancy weight, used for calculating the pregestational BMI, and history of adverse pregnancy. In addition, at enrollment, this information included blood pressure, height, and current weight used to calculate BMI and circumference during pregnancy and to analyze the full lipid profile (TG, total cholesterol, high-density lipoprotein cholesterol, and low-density lipid protein cholesterol) blood collection.

### 2.3. Eligibility Criteria

We excluded participants with pregestational diabetes mellitus (DM), hypertension, psychiatric disorders, chronic maternal diseases (kidney disease, heart disease, epilepsy, renal failure, etc.), congenital malformations, and multiple pregnancies. Subjects with imperfect data were also excluded.

### 2.4. MetS and Diagnosis Components

ATPIII, CDS, and IDF had published the diagnostic criteria for MetS, but there was no confirmed diagnostic gold standard. There are also no clear diagnostic criteria for the gestational metabolic syndrome. MS was diagnosed according to the classification by the Diabetes Branch of the Chinese Medical Association (CMA) [4]. Women with 3 or all of the following 4 components were diagnosed: (1) overweight or obesity (BMI ≥ 25 kg/m^2^); (2) high blood sugar; (3) hypertension; (4) lipid metabolism disorder. The maternal factors investigated were pre-BMI, anthropometric measurements, blood pressure (BP), and metabolic profile. GDM was diagnosed meeting one of the following standards: fasting glycemia ≥5.1 mmol/l; one-hour levels ≥10 mmol/l; two-hour levels ≥8.5 mmol/l, respectively, after a 75 g-OGTT. Hypertension was defined as follows: systolic blood pressure ≥140 mmHg or diastolic blood pressure ≥90 mmHg, or both, after 20 weeks of gestation, but before delivery or miscarriage on at least 2 occasions separated by at least 4 hours. Maternal pregnancy BMI was categorized into underweight (<18.5 kg/m^2^), normal weight (18.5–24.9 kg/m^2^), overweight or obesity (25.0–29.9 kg/m^2^, or ≥30 kg/m^2^) according to the World Health Organization BMI classification [5]. Fasting blood TG ≥ 1.7 mmol/L and (or) fasting blood HDL-C ≤ 1.0 mmol/L were diagnosed with hyperlipidemia [1].

### 2.5. Adverse Pregnancy Outcomes

Adverse pregnancy outcomes include maternal and fetal outcomes. Maternal pregnancy outcomes include miscarriage, preeclampsia, oligohydramnios, polyhydramnios, anemia, premature rupture of membranes, placental abruption, and preterm birth, and women with a history of adverse events during pregnancy, including previous miscarriage, fetal death, stillbirth, and fetal malformations. Low birth weight, macrosomia, fetal malformation death or death, fetal distress, and a low Apgar score (Apgar score ≤ 7 at 1 or 5 minutes) were defined as fetal outcomes.

### 2.6. Follow-Up

Follow-up was performed until the end of pregnancy (delivery or miscarriage). For women with GDM, the CDS-recommended protocol for maternal hyperglycemia control was followed. Diseases that occur during pregnancy are treated under the guidance of a professional doctor.

### 2.7. Statistical Analysis

Statistical analyses were done using Statistical Product and Service Solutions (SPSS), version 23.0 (IBM, Armonk, NY, USA). The Kolmogorov–Smirnov test was employed to determine the measurement data normality. Normally distributed continuous variables were analyzed using the *t*-test. The Mann–Whitney *U* test was used when the variable distribution was abnormal, and the *χ*^2^ test or Fisher's exact test was used to compare categorical variables. Through ROC curve analysis, the optimal cut-off points of maternal lipid profiles in prepregnancy and midpregnancy for predicting the metabolic syndrome in pregnancy were determined. Each optimal cutoff point was based on the maximum Youden Index (sensitivity + specificity − 1). AUC was calculated to evaluate the predictive powers. The confidence interval was set as 95% and the significance level was set at *P* < 0.05.

## 3. Results

Overall, 229 aged ≥ 35 and 536 aged 20-34 maternal women participated in this research (Table 1). The analysis in baseline characteristics revealed that history of adverse pregnancy, gravidity, and parity in the maternal age ≥35 group were significantly higher than those in the 20–34 maternal age group, and the difference had statistical significance (25.3% vs. 15.3%, *P* = 0.001; 2 (1, 2) vs. 1 (1, 1); 3 (2, 4) vs. 1 (1, 2), both *P* < 0.001).

BMI in the maternal age ≥35 group was higher than those in the 20–34 age group, and the difference had statistical significance (23.25 ± 3.34 vs. 22.15 ± 3.32, *P* < 0.001). The prevalence of overweight and obesity were more likely to happen in the maternal age ≥35 group than in the maternal age 20–34 group (23.58% vs. 16.30%, *P* = 0.012), and the prevalence of underweight was more likely to occur in the maternal age 20–34 group than the maternal age ≥35 group (5.52% vs. 2.18%, *P* = 0.001). The incidence of normal weight between the two groups has no statistical difference.

Met frequency was 9.6% in the maternal age ≥35 group, 5.4% in the maternal age 20–34 group (*P* = 0.027), and 6.7% in all pregnant women. Prevalence of metabolic syndrome components showed that GDM and MetS were more likely to happen in maternal age ≥35 group than in the maternal age 20–30 group (41.5% vs. 30.6%; *P* = 0.001, 9.6% vs. 5.4%, *P* = 0.027).

We found that women aged ≥35 years exhibited shorter gestational weeks than the younger controls (38.70 ± 1.65 vs. 39.17 ± 1.56, *P* < 0.001), and the birth weight in the maternal age ≥35 group was more than that in the maternal age 20–34 group (3310.05 ± 483.71 vs. 3232.00 ± 475.20, *P* = 0.039). The prevalence of macrosomia between the two groups has no statistical difference. (7.4% vs. 3.9%, *P* = 0.034). We also found that the GWG in the maternal age ≥35 group was less than those in the maternal age 20–34 group (11.23 ± 4.77 vs. 12.16 ± 4.72, *P* = 0.014).

From the second-trimester lipid profiles, TG and TC median levels were 1.08 mmol/L and 4.54 mmol/L, respectively (Table 2).

In the maternal age ≥35 group, the frequency of preterm labor was 22.7% and 6.7% (*P* = 0.024), and the frequency of eclampsia was 13.6% and 1.4% (*P* = 0.013) in the subgroups with and without the MetS. The frequency of preterm labor was 17.2% and 5.7% (*P* = 0.030) and the frequency of eclampsia was 27.6% and 2.0% (*P* < 0.001) in both subgroups with the maternal age 20–34 group. Results showed that macrosomia was more likely to happen in the maternal age ≥35 group than in the maternal age 20–34 group (7.0% vs. 4.1%; *P* = 0.034) (Table 3).

For preterm delivery and eclampsia, the relative risk at study participants are shown in Table 4. The risk for preterm delivery was added with increased BMI (RR = 1.082, 95% CI = 1.013–1.1568), hypertension (RR = 1.212, 95% CI = 1.049–1.399), and MetS (RR = 3.434, 95% CI = 1.020–1.340), but not with age, GDM, nor with hyperlipemia. The risk for eclampsia was increased with raised BMI (RR = 1.082, 95% CI = 1.026–1.1428), hypertension (RR = 1.800, 95% CI = 1.418–2.285), and MetS (RR = 1.252, 95% CI = 1.142–2.612), but not with age, GDM, nor with hyperlipemia.

In participants aged ≥35 years, we discovered that pre-BMI (OR 1.852, 95% CI 1.492–2.299) and the TC level (OR 2.509, 95% CI 1.551–4.060) were associated with an increased risk of MetS. In women aged 20–34 years, we observed that pre-BMI (OR 1.444, 95% CI 1.292–1.613), TG level (OR 1.499, 95% CI 1.058–2.124), LDL-C level (OR 1.847, 95% CI 1.059–3.222), and age (OR 1.300, 95% CI 1.061–1.592) were related to an increased risk of MetS (Table 5).

Pre-BMI predicting MetS in women aged ≥35 years had the largest AUC (AUC 0.925, 95% CI 0.885 to 0.965) and its optimal cutoff point was ≥24.998 kg/m^2^; the optimal cutoff points for TC (AUC 0.686, 95% CI 0.571–0.802) predicting MetS were ≥4.955 mmol/l. Pre-BMI predicting MetS had the largest AUC (AUC 0.890, 95% CI 0.834–0.945)). The optimal cutoff points were ≥1.075 mmol/L for TG predicting MetS and ≥2.745 mmol/L for LDL-C predicting MetS in women aged 20–34 years (Table 6).

## 4. Discussion

Older women are at an increased risk of adverse outcomes caused by the decay of reproductive function. There are several definitions to characterize MetS [6, 7]. In 2019, a study evaluated that the morbidity of MetS at 4 months of gestation was about 3.0% [8]. Another report demonstrated higher prevalence with 12.3% in women at the pregnancy stage of 14–16 weeks [9].

Analysis of adverse pregnancy outcomes showed that the incidence of GDM in women aged ≥35 years is higher. Considering this, our study suggested that an advanced maternal age accelerated the occurrence rate of adverse pregnancy outcomes [10, 11]. Elderly pregnant women have more attention to weight control during pregnancy. But we observed an increase in birth weight at advanced maternal age, indicating that women aged over 35 should be alarmed on pre-BMI and second-trimester lipid levels. We should also focus on GWG in pregnant women aged between 20 and 34.

In this chapter, we observed significant differences between the two groups regarding the kinds of adverse pregnancy outcomes. Some scholars also believe that there is insufficient evidence to prove whether an advanced maternal age is an independent direct risk factor for preterm birth and small-for-gestational-age birth [12–15]. We found that low levels of HDL-C at the midstage of pregnancy and hypertension were related to the incidence of spontaneous preterm deliveries, indicating that MetS should be traced closely [7, 16].

Our current study showed that pre-BMI, blood pressure (BP), and metabolic syndrome may be related to premature delivery and eclampsia. Given this, it is meaningful to have the necessary counseling and education about weight management and blood pressure control during pregnancy before conception [16]. The utility of the metabolic syndrome and diagnoses for predicting adverse pregnancy outcomes require detection.

Our study indicates that pre-BMI can predict MetS in pregnancy. Our findings suggested lipid profiles can predict MetS, TC in women with maternal age ≥35 years, and TG and LDL-C in maternal women aged between 20 and 34. Examining lipid profiles in pre-BMI and midtrimester can provide insight into the underlying mechanisms of MetS and contribute to a better understanding of the risk factors underlying each condition. Maternal obesity increases the risk of premature death and cardiovascular diseases. Pregnancy and early postpartum offer opportunities for interventions to identify obesity and reduce its adverse outcomes [17, 18].

## 5. Conclusion

MetS in pregnancy are more to occur in the maternal age ≥35 group than in the younger controls. MetS are related to the occurrence of preterm delivery and eclampsia; pre-BMI and TC can predict MetS in the maternal age ≥35 group. Advanced maternal age women should have more attention to weight control before pregnancy.

## Figures and Tables

**Table 1:** Study participants' characteristics.

Items	Group A (*n* = 229)	Group B (*n* = 536)	*P*-value
Age (years)	37.20 ± 2.08	29.94 ± 2.58	<0.001
History of adverse pregnancy, *n* (%)	58 (25.3)	82 (15.3)	0.001
Gravidity	2 (1.2)	1 (1.1)	<0.001
Parity	3 (2.4)	1 (1.2)	<0.001
BMI (kg/m^2^) in prepregnancy	23.25 ± 3.34	22.15 ± 3.32	<0.001
BMI groups			
Underweight, *n* (%)	5 (2.18)	46 (5.52)	0.001
Normal weight, *n* (%)	170 (74.24)	402 (75.19)	0.424
Overweight or obesity, *n* (%)	54 (23.58)	88 (16.30)	0.012
IVF-ET, *n* (%)	15 (6.55)	19 (3.51)	0.050
GWG (kg)	11.23 ± 4.77	12.16 ± 4.72	0.014
Gestational week	38.70 ± 1.65	39.17 ± 1.56	<0.001
Birth weight (g)	3310.05 ± 483.71	3232.00 ± 475.20	0.039
GDM, *n* (%)	95 (41.5)	165 (30.6)	0.001
Abnormal lipid metabolism, *n* (%)	82 (35.8)	167 (31.5)	0.121
Hyperlipemia, *n* (%)	14 (6.1)	40 (7.5)	0.309
MetS, *n* (%)	22 (9.6)	29 (5.4)	0.027

**Table 2:** Second-trimester lipid profiles by maternal age groups.

	Group A (*n* = 229)	Group B (*n* = 536)	*P-*value
TG	1.08 (0.74, 1.69)	0.90 (0.65, 1.35)	0.001
TC	4.54 (3.96, 5.21)	4.33 (3.82, 5.09)	0.029
HDL-C	1.66 (1.41, 1.94)	1.62 (1.39, 1.83)	0.068
LDL-C	2.27 (1.88, 2.86)	2.23 (1.83, 2.72)	0.341

**Table 3:** Pregnancy outcomes in maternal women with and without MetS.

	Number (%) of events						*P* value
	MetS in the maternal age 20–34 group (*n* = 229)			MetS in the maternal age 20–34 group (*n* = 536)			
	Yes (%) (*n* = 22)	No (%) (*n* = 207)	*P-*value	Yes (%) (*n* = 29)	No (%) (*n* = 507)	*P* value
Miscarriage	0 (0)	4 (1.9)	0.666	0 (0)	3 (0.6)	0.846	0.124
Preterm labor	5 (22.7)	14 (6.7)	0.024^*∗*^	5 (17.2)	29 (5.7)	0.030^*∗*^	0.205
Placental abruption	0 (0)	2 (0.7)	0.817	1 (3.4)	4 (0.8)	0.224	0.649
Eclampsia	3 (13.6)	3 (1.4)	0.013^*∗*^	8 (27.6)	10 (2.0)	<0.001^*∗*^	0.389
PPROM	3 (13.6)	18 (8.7)	0.327	2 (6.9)	47 (9.3)	0.494	0.544
Postpartum hemorrhage	5 (22.7)	52 (25.1)	0.519	7 (24.1)	118 (23.3)	0.533	0.352
Oligohydramnios	1 (4.5)	2 (1.0)	0.262	0 (0)	7 (1.4)	0.676	0.514
Polyhydramnios	1 (4.5)	0 (0)	0.904	0 (0)	2 (0.4)	0.895	0.657
Low birthweight infant	2 (9.1)	6 (2.9)	0.173	2 (6.9)	25 (4.9)	0.437	0.231
Macrosomia	1 (4.5)	15 (7.2)	0.531	0 (0)	21 (4.1)	0.304	0.034^*∗*^
Low Apgar scores (Apgar score at 1 min or 5 min ≤ 7)	1 (4.5)	4 (1.9)	0.399	0 (0)	15 (3.0)	0.429	0.417
Stillbirth and fetal deformity	1 (4.5)	4 (1.9)	0.399	2 (6.9)	9 (1.8)	0.115	0.254

**Table 4:** The relative risk for study participants at preterm delivery.

	Preterm delivery			
		RR	95% CI	*P* value
Age ≥ 35	*n* = 229, *N* = 19, 8.3%	1.021	0.977, 1.608	0.205
BMI ≥ 25	*n* = 141, *N* = 18, 12.8%	1.082	1.013, 1.156	0.004
GDM	*n* = 251, *N* = 23, 9.3%	1.037	0.991, 1.084	0.054
Hypertensive	*n* = 54, *N* = 12, 22.2%	1.212	1.049, 1.399	<0.001
Hyperlipemia	*n* = 249, *N* = 17, 8.5%	0.998	0.958, 1.040	0.536
MetS	*n* = 51, *N* = 10, 19.6%	1.169	1.020, 1.340	0.002

**Table 5:** Logistic regression analysis of potential effective factors on MetS in the two groups.

	OR	95% CI	*P* value
Maternal age ≥35 group (*n* = 229)			
Pre-BMI	1.852	1.492–2.299	<0.001
TC	2.509	1.551–4.060	<0.001

Maternal age 20–34 group (*n* = 536)			
Pre-BMI	1.444	1.292–1.613	0.023
TG	1.499	1.058–2.124	0.031
LDL-C	1.847	1.059–3.222	<0.001
Age	1.300	1.061–1.592	0.011

**Table 6:** Optimal cut-off points of pre-BMI and maternal trimester lipids for predicting metabolic syndrome in pregnant women.

	AUC (95% CI)	Sensitivity (%)	Specificity (%)	Youden index	Cut-off point
Maternal age ≥35 group (*n* = 229)					
Pre-BMI (kg/m^2^)	0.925 (0.885–0.965)	90.9	83.6	0.745	24.998
TC (mmol/l)	0.686 (0.571–0.802)	63.6	71.5	0.351	4.955

Maternal age 20–34 group (*n* = 536)					
Pre-BMI (kg/m^2^)	0.890 (0.834–0.945)	86.2	88.0	0.742	25.043
TG (mmol/l)	0.766 (0.685–0.847)	82.8	64.7	0.475	1.075
LDL-C (mmol/l)	0.741 (0.649–0.834)	71.4	78.7	0.501	2.745

## Data Availability

The datasets used and analyzed during the current study are available from the corresponding author upon request.
